# A Dynamic Adaptive Weighted Differential Evolutionary Algorithm

**DOI:** 10.1155/2022/1318044

**Published:** 2022-06-29

**Authors:** Kaijun Wu, Zhengnan Liu, Ning Ma, Dicong Wang

**Affiliations:** ^1^School of Electronic and Information Engineering, Lanzhou Jiaotong University, Lanzhou 730070, China; ^2^Department of Intelligence and Computing, Tianjin University, Tianjin 300354, China

## Abstract

This study proposed a dynamic adaptive weighted differential evolution (DAWDE) algorithm to solve the problems of differential evolution (DE) algorithm such as long search time, easy stagnation, and local optimal solution. First, adaptive adjustment strategies of scaling factor and crossover factor are proposed, which are utilized to dynamically balance the global and local search, and avoid premature convergence. Second, an adaptive mutation operator based on population aggregation degree is proposed, which takes population aggregation degree as the amplitude coefficient of the basis vector to determine the influence degree of the optimal individual on the mutation direction. Finally, the Gauss perturbation operator is introduced to generate random disturbance and accelerate premature individuals to jump out of the local optimum. The simulation results show that the DAWDE algorithm can obtain better optimization results and has the characteristics of stronger global optimization ability, faster convergence, higher solution accuracy, and stronger stability compared with other optimization algorithms.

## 1. Introduction

The differential evolution (DE) algorithm is an optimization algorithm based on the theory of modern intelligence [1]. It was first proposed by American scholars Rainer Storn and Kenneth Price in 1995 to solve the Chebyshev inequality [2]. The DE algorithm solves the problem by simulating the biological evolution of the survival of the fittest [3]. Superior to the traditional optimization algorithm such as the method based on calculus [4] and the exhaustive method [5], the DE algorithm uses its unique memory ability to track the current search situation and adjust the search strategy at the same time. It has high robustness and strong global convergence ability and can effectively deal with complex problems that are difficult to be solved by the traditional optimization algorithms. In addition, the DE algorithm is not limited by the nature of the problem, for example, derivatives are not required as auxiliary information and are not constrained by search space constraints (such as continuous differentiability and single peak) [6–9]. It is widely used in constrained optimization calculation, neural network optimization, filter design, etc.

In recent years, the DE algorithm is widely used and is also a concern by scholars around the world. Wang et al. [10] proposed a generalized reverse differential evolution algorithm, which introduced acceleration and migration operations in DE. The acceleration operation used gradient information to lead the optimal individual to a better area, and when the dispersion of the population is lower than a certain threshold, the migration operation is used to regenerate new individuals in the vicinity of the optimal individual and replace the old individual, thereby maintaining the diversity of the population and preventing the algorithm from falling into local optimum to a certain extent. Chiou et al. [11] proposed a variable scaling hybrid differential evolution (VSHDE) algorithm, which does not need to select the type of mutation operation, but selects the appropriate mutation operator for DE from a variety of mutation operators in real time to speed up the optimization process of the algorithm. Compared with the random scale factor, the algorithm has a great improvement in performance. Qin et al. [12] proposed the SaDE algorithm to adaptively adjust *F* and *CR* based on the experience of early evolution to generate high-quality solutions. Brest et al. [13] proposed a differential evolution (JDE) algorithm for adaptive control parameters and introduced new control parameters to adjust the values of *F* and *CR* through a comparative study of numerical benchmark problems. Zhang et al. [14] introduced a new mutation strategy “DE/current-to-pbest” to improve the optimization performance of the algorithm and proposed an adaptive differential evolution (JADE) algorithm with optional external archiving. Hou Ying et al. [15] introduced a dynamic multiobjective differential evolution algorithm, based on the information on evolution progress (DMODE-IEP), which is developed to improve the optimization performance. The information of evolution progress, using the fitness values, is proposed to describe the evolution progress of MODE, and the dynamic adjustment mechanisms of evolution parameter values, mutation strategies, and selection parameter values based on the information on evolution progress are designed to balance the global exploration ability and the local exploitation ability.

Aiming at the problems of long search time, easy stagnation, and easy to fall into the local optimal solution of the differential evolution algorithm [16], this study proposes a dynamic adaptive weighted differential evolution (DAWDE) algorithm on the basis of the above several improved algorithms. We select several typical benchmark functions to test [16, 17]. The test results show that the DAWDE algorithm has relatively strong global optimization ability, strong convergence performance, and is not easy to fall into the local optima. The global optimal values obtained are all near or equal to the given optimal value.

## 2. DE Algorithm

The DE algorithm is an algorithm based on group evolution, which can not only memorize the optimal solution of individuals but also has the characteristics of information sharing within the population. It is a method of optimization used in symmetrical optimization problems and also in problems that are not even continuous, and are noisy and change over time [18]. The essence is a greedy genetic algorithm based on actual number coding and with the idea of preserving optimality [19].

In the DE algorithm, each population is composed of *NP* individuals, which is expressed as follows: *X*^0^={*x*_1_^0^, *x*_2_^0^,…, *x*_*NP*_^0^}, where *NP* is the population size; each individual is used to represent the solution of the problem, which is expressed as follows: *x*_*i*_^0^={*x*_*i*,1_^0^, *x*_*i*,2_^0^,…, *x*_*i*,*D*_^0^}, where *D* is the dimension of the solution, *x*_*i*_^0^ is the i^th^ individual in the 0^th^ generation population, and *x*_*i*,*j*_^0^ is the j^th^ component of the i^th^ individual in the 0^th^ generation population. The main operation steps of the algorithm are as follows.

### 2.1. Initialization

(1) $$\begin{array}{c} x_{i,j}^{0}=x_{i,j}^{\min}+\text{rand}\left(0,1\right)\cdot \left(x_{i,j}^{\max}-x_{i,j}^{\min}\right), \end{array}$$

where *x*_*i*,*j*_^max^ and *x*_*i*,*j*_^min^ represent the upper and lower bounds of the j^th^ dimension optimization, respectively, and rand(0,1) represents a random number in the interval [0,1].

### 2.2. Mutation

The DE algorithm realizes individual mutation through the difference strategy, randomly selects two different individuals to scale their vector differences, and performs vector synthesis with the individual to be mutated to generate corresponding mutated intermediate individuals. The most commonly used strategy in mutation operation is DE/rand/1/bin, and the specific expression is as follows:

(2) $$\begin{array}{c} v_{i}^{g+1}=x_{r1}^{g}+F\cdot \left(x_{r2}^{g}-x_{r3}^{g}\right), \end{array}$$

where *i* ≠ *r*1 ≠ *r*2 ≠ *r*3, and g is the current iteration number, that is, the g^th^ generation. *F* is the scaling factor. The smaller the *F* is, the stronger the local search ability is; the larger the *F* is, the more it can jump out of the local area.

### 2.3. Crossover

The DE uses the original individual *x*_*i*_^*g*^ and the mutant intermediate individual *v*_*i*_^*g*+1^ to cross to generate a new individual *u*_*i*_^*g*+1^, and determines whether the new individual gene is provided by the original individual or the mutant intermediate individual according to whether the conditions are met. The crossover operation is as follows:

(3) $$\begin{array}{c} u_{i,j}^{g+1}=\left\{\begin{array}{c} v_{i,j}^{g+1},\text{ if rand}\left(0,1\right)\leq CR\text{ or }j=j_{\text{rand}}\\ x_{i,j}^{g},\text{ otherwise} \end{array}\right., \end{array}$$

where *CR* is the crossover probability, and *j*_rand_ is a random integer on [1,  *D*]. *j*=*j*_rand_ means *j* is randomly selected so that one gene in *u*_*i*_^*g*+1^ is contributed by *v*_*i*_^*g*+1^ to ensure the generation of new individuals, and the rest of the genes are determined by the crossover probability factor *CR*. The larger *CR* is, the more *v*_*i*_^*g*+1^ contributes to *u*_*i*_^*g*+1^, which is conducive to improving local development capabilities; the smaller *CR* is, the more *x*_*i*_^*g*^ contributes to *u*_*i*_^*g*+1^, which is conducive to improving global search capabilities [20].

### 2.4. Selection

The DE algorithm adopts a greedy strategy when selecting operations, and only those with better fitness values are selected for the next generation. The selection operation is as follows:

(4) $$\begin{array}{c} x_{i,j}^{g+1}=\left\{\begin{array}{c} u_{i,j}^{g+1},f\left(u_{i,j}^{g+1}\right)<f\left(x_{i,j}^{g}\right)\\ x_{i,j}^{g},f\left(u_{i,j}^{g+1}\right)\geq f\left(x_{i,j}^{g}\right) \end{array}.\right. \end{array}$$

## 3. Dynamic Adaptive Weighted Differential Evolution (DAWDE) Algorithm

### 3.1. Scale Factor *F* Adaptive Adjustment Strategy

According to formula (2), the scaling factor *F* in the mutation operation is an important parameter to control the diversity and convergence of the population, and it determines the magnification ratio of the deviation vector. The smaller the value of *F* is, the smaller the group difference is, which will speed up the algorithm convergence and also lead to the local convergence of the algorithm, while the larger the value *F* is, it will help the algorithm to jump out of the local optimal solution, but it will reduce the convergence speed. In order to balance the local and global search and maintain a fast convergence rate, an adaptive adjustment strategy is proposed as follows:

(5) $$\begin{array}{c} F=F_{\text{max}}-\left(F_{\max}-F_{\min}\right){\left(\frac{g}{G}\right)}^{2}, \end{array}$$

where *F*_max_ is the maximum value of the scaling factor, which is 0.9, and *F*_min_ is the minimum value of the scaling factor, which is 0.2, *g* is the current iteration number, that is, the g^th^ generation, and *G* is the maximum iteration number.

### 3.2. Dynamic Adjustment Strategy of Crossover Probability Factor *CR*

The crossover probability factor *CR* determines whether the new individual gene is provided by the original individual or the mutant intermediate individual, that is, the degree of participation of each dimension of individual parameters in the crossover. The smaller the *CR* is, the better individuals are retained, and the faster the algorithm converges, but it is easy to fall into the local optimum value. The larger *CR* is, the higher the diversity of the population is, and the better the global search ability is, but the convergence speed of the algorithm will decrease accordingly. In this study, a dynamic adaptive crossover factor is adopted, and *CR* is set as a dynamic adaptive function that continuously oscillates in [0,1] and is updated every 50 generations, so that the constant change in *CR* can make the new individual randomly inherit the mutant individual or parent generation of individual genes, jumping out of the local optimal solution. The value is as follows:

(6) $$\begin{array}{c} CR_{\text{g}}=\left\{\begin{array}{c} \frac{1+\cos\;g}{2},\mathrm{mod}\left(g,50\right)=0\\ CR_{g-1},\text{otherwise} \end{array},\right. \end{array}$$

where *CR*_*g*_ is the value of *CR* of the g^th^ generation, *CR*_*g*−1_ is the value of *CR* of the g-1^th^ generation, and mod(*g*, 50)=0 is to be updated every 50 generations.

### 3.3. Adaptive Mutation Operator Based on Population Aggregation Degree

In the later stage of the iteration of the DE algorithm, the difference between individuals of the population decreases, the diversity decreases, finally, the aggregation phenomenon is formed, and the definition of population aggregation degree is proposed.

Assuming that the size of the group is *NP*, the particle dimension is *D*, *x*_*i*,*j*_ is the individual vector of individual *x* on the j^th^ dimension, and $\bar{x_{j}}$ is the average value of the individual vector particles of the population on the jth dimension, then the population aggregation degree can be defined as follows:

(7) $$\begin{array}{c} C=\sum_{j=1}^{D}\sum_{i=1}^{NP}\left|x_{i,j}-\bar{x_{j}}\right|. \end{array}$$

The smaller the population aggregation degree *C* is, the smaller the individual differences of the population is, and the higher the aggregation degree is; on the contrary, it means that the population individuals are scattered and the population diversity is good. Therefore, the population aggregation degree *C* can well describe the aggregation degree of population individuals. In this study, *C* takes [0.05, 0.95].

The main purpose of improving the DE algorithm is to balance the global exploration ability and local development ability of the algorithm. The standard DE algorithm adopts a random selection mutation strategy, expressed as DE/rand/1, which is beneficial to improve the diversity of mutation and global exploration ability, but the randomness interferes with the evolution direction in a large range, with great blindness and uncertainty, which may lead to algorithm premature and limited convergence speed. While DE/best/1 uses the optimal individual as the mutation base to ensure the optimal direction of evolution and local development ability, the optimal individual may be the local optimal individual. If the population keeps evolving in this direction, it is very likely to fall into the local optimum. The mutation strategies DE/best/1 and DE/rand/1 of the standard differential evolution algorithm are

(8) $$\begin{array}{c} \left\{\begin{array}{c} v_{i}^{g+1}=x_{\text{best}}^{g}+F\cdot \left(x_{r1}^{g}-x_{r2}^{g}\right)\\ v_{i}^{g+1}=x_{\text{r}3}^{g}+F\cdot \left(x_{r4}^{g}-x_{r5}^{g}\right) \end{array}\right., \end{array}$$

We carry out the weighted combination to propose a new weighted dynamic mutation strategy as follows:

(9) $$\begin{array}{c} v_{i}^{g+1}=C\cdot \left[x_{\text{best}}^{g}+F\cdot \left(x_{r1}^{g}-x_{r2}^{g}\right)\right]+\left(1-C\right)\cdot \left[x_{r3}^{g}+F\cdot \left(x_{r4}^{g}-x_{r5}^{g}\right)\right], \end{array}$$

where *i*, *r*1, *r*2, *r*3, *r*4, *r*5 are random integers on [1, *NP*] and are not equal to each other. *x*_best_^*g*^ is the optimal individual of the g^th^ generation population.

According to formula (5), the population aggregation degree *C*, as the weight of the influence of the optimal individual on the variation direction, is a monotonically increasing function; then, 1 − *C* is a monotonically decreasing function. After weighted merging, in the early stage of optimization, the amplitude coefficient of *x*_best_^*g*^+*F* · (*x*_*r*1_^*g*^ − *x*_*r*2_^*g*^) is small, and the amplitude coefficient of *x*_*r*3_^*g*^+*F* · (*x*_*r*4_^*g*^ − *x*_*r*5_^*g*^) is large, focusing on global exploration, and in the later stage of optimization, the amplitude coefficient of *x*_best_^*g*^+*F* · (*x*_*r*1_^*g*^ − *x*_*r*2_^*g*^) increases, and the amplitude coefficient of *x*_*r*3_^*g*^+*F* · (*x*_*r*4_^*g*^ − *x*_*r*5_^*g*^) reduces, focusing on local development, so that the algorithm takes into account the global search ability and local development ability at the same time, which is not only beneficial to the diversity of the population but also improves the convergence speed of the algorithm.

### 3.4. Disturbance Dimensional Mutation to Get Out of Premature

When solving high-dimensional complex function problems, problems such as falling into local optimum will generally occur in the later stage of the DE algorithm. In order to describe the state of the population, the following premature definitions are given as follows:

Let *Q* be the precocious period, and if *M*od(g,Q)=0 and the difference between the current fitness value and the fitness value before *Q* generations is extremely small, that is,

(10) $$\begin{array}{c} \left|f_{\text{best}}\left(\text{g}\right)-f_{\text{best}}\left(g-Q+1\right)\right|\leq \delta , \end{array}$$

the individual is said to be premature in the *Q* generation iteration. Among them, *f*_best_(*g*) is the optimal fitness value of the g^th^ generation, and *δ* is the premature test threshold and takes *δ*=1*E* − 6.

If it is judged by the above formula that the algorithm has been premature, the dimensional mutation is carried out, and the mutation strategy is as follows:

(11) $$\begin{array}{c} x_{i,j}^{g}=C\cdot x_{\text{best},j}^{\text{g}}+\left(1-C\right)\cdot x_{r1,j}^{g}+\alpha \left(x_{r2,j}^{g}-x_{r3,j}^{g}\right), \end{array}$$

where the weighting coefficient *C* is the same as formula (5), *α*=*F*(1+0.5*η*) is the acceleration random disturbance coefficient, *η* is a random variable obeying the distribution Gauss(0,1), and *x*_best_^*g*^ is the optimal individual of the g^th^ generation on the j^th^ dimension.

It can be seen from formula (9) that the dimensional mutation strategy consists of two parts, the *C* · *x*_best,*j*_^g^+(1 − *C*) · *x*_*r*1,*j*_^*g*^ part is composed of the optimal individual and the weight of random individuals, and the information of the optimal individual is used to guide other individuals to evolve toward the optimization direction; the *α*(*x*_*r*2,*j*_^*g*^ − *x*_*r*3,*j*_^*g*^) part is the accelerated random disturbance vector; and since the individual has fallen into the local optimum, disturbance mutation is randomly generated, which accelerates the individual to jump out of the local optimum and guides the individual to explore the global.

### 3.5. Algorithm Steps

**Step 1 .**

Initialization parameters: population size *NP*, solution dimension *D*, maximum evolutionary generation *G*, upper bound of individual variables *x*_*i*,*j*_^max^, lower bound of individual variables *x*_*i*,*j*_^min^, maximum sum of scaling factors *F*_max_, minimum sum of scaling factors *F*_min_, premature generation *Q*, and premature test threshold *δ*.

**Step 2 .**

Initialize the population, calculate the fitness value of each individual, and find out the individual of optimal fitness value *x*_best_ and the corresponding optimal fitness value *f*_best_.

**Step 3 .**

Calculate *F*, *CR*, and *C*, according to formulas (5)–(7).

**Step 4 .**

Mutation operations. The variant individual *v*_i_^*g*+1^ is obtained according to formula (9).

**Step 5 .**

Crossover operations. A new test individual *u*_*i*,*j*_^*g*+1^ is obtained according to the formula (3).

**Step 6 .**

Selection operations. The next generation *x*_*i*,*j*_^*g*+1^ is obtained from the formula (4).

**Step 7 .**

Update the local and global optimal values.

**Step 8 .**

Check for premature. If *Mod*(*g*, *Q*)=0 and |*f*_best_(g) − *f*_best_(*g* − *Q*+1)| ≤ *δ*, calculate a new individual *x*_*i*,*j*_^*g*^ according to formula (11), and update the optimal value to jump out of the local optimum.

**Step 9 .**

Repeat Steps 4–8.

**Step 10 .**

If the maximum number of iterations *G* is not reached, go to Step 3; otherwise, continue.

**Step 11 .**

Output the optimal value *x*_best_ and *f*_best_.

## 4. Experimental Results

### 4.1. Test Functions and Comparison Algorithm

In order to verify the effectiveness of the algorithm, this algorithm is compared with the standard DE/rand/1, SaDE algorithm, and JADE algorithm. All algorithms are independently run 20 times on 8 typical test functions. The test functions are shown in Table 1. Their global optimal values are all 0. According to the obtained optimal solution and convergence curve, the performances of each algorithm in terms of convergence speed, optimal solution accuracy, and robustness are compared.

The simulation experiment is programmed with MATLAB R2016a software, and the experimental configuration is Intel(R) Core(TM) i5-6300HQ CPU@2.30 GHz. The basic parameters of the algorithm are set as follows: *NP*=50, *F*_max_=0.9, *F*_min_=0.2, *Q*=10, and *δ*=1E − 6, and the compared algorithm DE/rand/1, SADE, and JADE parameter settings are the same as the original. In order to examine the comprehensive performance of the algorithm, considering the dimension *D*=30 and *D*=50 two cases, for the sake of fairness, the maximum number of iterations of all algorithms is 2000, and the algorithm is independently run 20 times.

### 4.2. Results and Analysis

The minimum value, average optimal value, and standard deviation of the solution results are shown in Table 2.

It can be seen from the analysis that the DAWDE algorithm can achieve better optimization results than the other four algorithms on the 8 test functions regardless of whether the dimension is 30 or 50. By comparing the best value, mean optimal value, and standard deviation, it can be seen that the DAWDE algorithm has strong global optimization ability and has great advantages compared with other algorithms in terms of convergence accuracy, convergence ability, and stability. The optimization performance of the DAWDE algorithm will not decrease due to the increase in the complexity of the function, which shows that the algorithm has high scalability, and it can be concluded from the standard deviation that the stability of the algorithm is strong. Compared with the other four algorithms, the theoretical optimal value of 0 cannot be obtained in 30 dimensions, and as the function becomes more complex, the optimal value converged by the algorithm deviates from the theoretical optimal value. It can be seen from the standard deviation that the stability of the other four algorithms in optimizing high-dimensional complex functions is also poor, and with the increase in the dimension, the evolutionary ability decreases to varying degrees.

Figures 1–8 show the fitness value convergencecurvesof the 5 algorithmstested for 8 functions. When we analyzedeach set of figures indetail, it can be seen from Figures 1(a) and 1(b) that for the function *f*_1_, although all the five algorithms can reach the theoretical optimal value of 0, the DAWDE algorithm has already converged to the optimal value before the 10^th^ generation, which is the fastest among these algorithms. The other four algorithms all have stagnation to a certain extent. According to Figures 2(a) and 2(b), when the dimension is 30, the DAWDE algorithm gets the optimal value before the fifth generation, whereas other functions get the optimal value after the fifth generation. When the dimension is 50, the DAWDE algorithm and the JDE algorithm both perform well on *f*_2_, and the other three functions all fall into local optimum during the convergence process. It can be seen from Figures 3(a) and 3(b) that the DAWDE algorithm converges to the optimal value of 0 very quickly on *f*_3_, while the DE algorithm and the JDE algorithm perform slightly worse. In 30 and 50 dimensions, the DE algorithm and the JDE algorithm are optimized in about 400^th^ generation and 1000^th^ generation, respectively. The JADE algorithm and the SaDE algorithm perform even worse, failing to get the optimal value and falling into the local optimum. As can be seen from Figures 4(a) and 4(b), for the function *f*_4_, the DAWDE algorithm converges faster than the other algorithms. Figures 5(a) and 5(b) show that, for the function *f*_5_, when the dimension is 30, the DAWDE algorithm gets the optimal value before the 10^th^ generation, whereas other functions get the optimal value after the 100^th^ generation. When the dimension is 50, the convergence of the DAWDE algorithm is still very fast, but other algorithms are affected by the increase in dimension, and the optimal is not reached until 200 generations later. It can be seen from Figures 6(a) and 6(b) that for the function *f*_6_, the algorithms DE and SADE both fall into local optimum, and the solution accuracy is poor. As can be seen from Figures 7(a) and 7(b), for the function *f*_7_, although all five algorithms can obtain the optimal value, the curve convergence speed of the DAWDE algorithm is significantly faster than that of the other four algorithms. Figures 8(a) and 8(b) show that, for the function *f*_8_, when the other four algorithms fall into the local optimum, the DAWDE algorithm can still quickly obtain the optimum value, indicating that it has the ability to judge and jump out of premature. Comparing the 30-dimensional and 50-dimensional figures, it can be seen that although the spatial dimension has increased, the optimization ability of the DAWDE algorithm has not been significantly reduced. In contrast, the optimization capabilities of the other four algorithms have decreased to varying degrees, which proves that the DAWDE algorithm not only adapts to the low-dimensional search space but also meets the requirements of high-dimensional search space. To sum up, the DAWDE algorithm performs well in the early stage of optimization, and the convergence speed is very fast. The optimal value can be obtained around the 20^th^ generation, and it is not affected by dimensions and has strong stability. Compared with DAWDE, the other four algorithms have a slower convergence speed and worse solution accuracy, and the more complex the function is, the more the objective function value deviates from the theoretical optimal value.

## 5. Conclusions

In this study, a dynamic adaptive weighted differential evolution (DAWDE) algorithm is proposed to solve the problems of long search time, easy stagnation, and easy to fall into local optimal solution when a differential evolution algorithm solves high-dimensional complex optimization problems. The improved algorithm includes adaptive optimization scaling factor and crossover factor, proposes an adaptive mutation operator based on the aggregation degree of the population, and adopts a random dimensional mutation and disturbance strategy. The algorithm dynamically balances the global exploration ability and local development ability of the algorithm. The simulation results show that the DAWDE algorithm can obtain better optimization results than other optimization algorithms on the 8 test functions. Regardless of the dimension, it has the characteristics of strong optimization ability, fast convergence, high solution accuracy, and strong stability, which provides a choice for solving complex high-dimensional optimization problems and also provides algorithm support for practical application research in the future [17].

## Figures and Tables

**Figure 1:** Convergence curve of *f*_1_. (a) 30 dimensions. (b) 50 dimensions.

**Figure 2:** Convergence curve of *f*_2_. (a) 30 dimensions. (b) 50 dimensions.

**Figure 3:** Convergence curve of *f*_3_. (a) 30 dimensions. (b) 50 dimensions.

**Figure 4:** Convergence curve of *f*_4_. (a) 30 dimensions. (b) 50 dimensions.

**Figure 5:** Convergence curve of *f*_5_. (a) 30 dimensions. (b) 50 dimensions.

**Figure 6:** Convergence curve of *f*_6_. (a) 30 dimensions. (b) 50 dimensions.

**Figure 7:** Convergence curve of *f*_7_. (a) 30 dimensions. (b) 50 dimensions.

**Figure 8:** Convergence curve of *f*_8_. (a) 30 dimensions. (b) 50 dimensions.

**Table 1:** Test functions.

Test functions	Formula	Initial range
Sphere	*f*_1_(*x*)=∑_*i*=1_^*n*^*x*_*i*_^2^	[−100, 100]
Schwefel's problem 2.2	*f*_2_(*x*)=∑_*i*=1_^*n*^|*x*_*i*_|+∏_*i*=1_^*n*^|*x*_*i*_|	[−10, 10]
Schwefel's problem 1.2	*f*_3_(*x*)=∑_*i*=1_^*n*^(∑_*j*=1_^*i*^*x*_*j*_)^2^	[−10, 10]
Ackley	$f_{4}\left(x\right)=-20\;\exp\left(-0.2\sqrt{\sum_{i=1}^{n}x_{i}^{2}}\right)-\exp\left(1/n\sum_{i=1}^{n}\cos\left(2\pi x_{i}\right)\right)+20+e$	[−32, 32]
Griewank	$f_{5}\left(x\right)=1/4000\sum_{i=1}^{n}x_{i}^{2}-\prod_{i=1}^{n}\cos\left(x_{i}/\sqrt{i}\right)+1$	[−600, 600]
Rastrigin	*f*_6_(*x*)=∑_*i*=1_^*n*^[*x*_*i*_^2^ − 10 cos(2*πx*_*i*_)+10]	[−5.12, 5.12]
Rosenbrock	*f*_7_(*x*)=∑_*i*=1_^*n*^[100(*x*_*i*+1_ − *x*_*i*_)^2^+(*x*_*i*_ − 1)^2^]	[−10, 10]
Schaffer	$f_{8}\left(x\right)=\sum_{i=1}^{n-1}\left[0.5+\sin^{2}\sqrt{x_{i}^{2}+x_{i+1}^{2}}-0.5/1+0.001{\left(x_{i}^{2}+x_{i+1}^{2}\right)}^{2}\right]$	[−100, 100]

**Table 2:** Test function optimization results of 30 dimensions and 50 dimensions.

*f*	Algorithm	30 dimensions			50 dimensions		
		Best	Mean	Std	Best	Mean	Std
*f*_1_	DE	5.34E-29	8.37 E+02	5.30 E+03	3.73E-13	2.08E-03	1.09 E+04
	SaDE	5.01E-28	8.90 E+02	5.05 E+03	1.28E-14	3.13 E+03	1.41 E+04
	JDE	1.34E-39	4.67 E+02	3.38 E+03	1.70E-26	1.61 E+03	8.88 E+03
	JADE	1.62×E-04	9.34×E-03	8.86×E-03	1.94×E-01	9.68 E+08	8.20 E+10
	DAWDE	0	0	0	0	0	0

*f*_2_	DE	4.94E-16	9.68 E+08	8.20 E+10	4.69E-09	1.27 E+20	1.19 E+22
	SaDE	6.99E-17	1.99 E+08	4.78 E+09	1.96E-09	7.31 E+17	2.26 E+19
	JDE	1.55E-24	2.53 E+05	1.08 E+07	1.22E-16	2.79 E+17	1.24 E+19
	JADE	6.02E-03	2.69E-02	1.51E-02	7.10E-01	1.54	6.23E-01
	DAWDE	0	0	0	0	0	0

*f*_3_	DE	4.70E-05	2.66E-01	1.02 E+02	7.54E-01	1.30 E+02	3.08 E+02
	SaDE	1.34 E+02	2.28 E+02	1.17 E+02	1.12 E+03	1.14 E+03	1.17 E+02
	JDE	3.61E-03	21.96	78.85	1.66	1.02 E+02	2.62 E+02
	JADE	1.68 E+02	2.49 E+02	31.64	5.12 E+02	7.77 E+02	1.01 E+02
	DAWDE	0	0	0	0	0	0

*f*_4_	DE	7.99E-15	1.16	3.65	1.15E-14	1.19	3.67
	SaDE	1.42E-14	1.14	3.63	1.95E-08	2.14	4.92
	JDE	7.99E-15	0.91	3.18	2.22E-14	1.27	3.8
	JADE	7.12E-05	78.42E-01	1.11E-03	4.36E-03	1.04	0.79
	DAWDE	8.88E-16	8.88E-16	0	8.88E-16	8.88E-16	0

*f*_5_	DE	0	7.52	46.54	2.41E-13	19	97.45
	SaDE	0	8.2	47.04	1.55E-14	26.69	1.15 E+02
	JDE	0	4.91	31.05	0	9.96	58.53
	JADE	5.03 E+02	2.52 E+03	5.56 E+02	8.98 E+02	4.19 E+03	9.60 E+02
	DAWDE	0	0	0	0	0	0

*f*_6_	DE	12.6	1.55 E+02	65.38	30.94	3.04 E+02	1.20 E+02
	SaDE	20.97	68.1	58.01	1.40 E+02	2.26 E+02	95.21
	JDE	0	27.37	61.39	1.40E-09	78.14	1.24 E+02
	JADE	5.11 E+02	1.95 E+03	9.81 E+02	1.21 E+02	1.43 E+03	1.03 E+03
	DAWDE	0	0	0	0	0	0

*f*_7_	DE	20.04	2.37 E+04	2.07 E+05	44.01	6.51 E+04	4.65 E+05
	SaDE	25.26	1.99 E+04	1.47 E+05	45.59	1.21 E+05	6.48 E+05
	JDE	17.92	7.02 E+03	7.08 E+04	27.73	3.78 E+04	2.67 E+05
	JADE	2.54	11.71	5.89	55.52	1.18 E+02	31.44
	DAWDE	0	0	0	0	0	0

*f*_8_	DE	10.47	12.04	0.5	19.52	21.72	0.6
	SaDE	6.32	8.42	1.63	16.17	18.21	1.57
	JDE	1.07	3.88	3.38	3.29	9.6	5.48
	JADE	0.15	0.48	0.14	1.87	2.93	0.35
	DAWDE	0	0	0	0	0	0

## Data Availability

The data used to support the findings of this study are available from the corresponding author upon request.
